This article has been retracted.

# The analysis of credit governance in the digital economy development under artificial neural networks

**DOI:** 10.1016/j.heliyon.2024.e39286

**Published:** 2024-10-11

**Authors:** Zhenzhen Huang, Zhiming Xu, Xiangyu Wang, Zhaoyi Xu

**Affiliations:** a School of Economics and Trade, Hunan University, Changsha, 410079, China; b Business School, Imperial College London, London, SW7 2BX, UK; c School of Economics and Management, Tsinghua University, Beijing, 100084, China

**Keywords:** Digital economy, Internet of things, Credit governance, Long short-term memory, Adaptive mechanisms

## Abstract

This paper aims to provide new avenues for innovation in credit governance in the digital economy to provide more reliable credit evaluation solutions for financial, commercial, and social interactions. This paper integrates the potential value of Internet of Things (IoT) technology in credit governance and proposes a credit governance method that utilizes IoT data and an improved Long Short-Term Memory model. The proposed model introduces an adaptive mechanism to monitor changes in data in real-time and automatically adjust network parameters to improve the model performance. Experimental validation is conducted on the University of California Irvine dataset. It is found that the proposed model performs well in terms of accuracy, F1 value, and Area Under the Curve value, with values of 0.9, 0.91, and 0.94, respectively. This indicates that the proposed model has higher classification accuracy and performance in classification tasks while maintaining efficient training time. This indicates that the presented method has potential application prospects in credit governance research.

## 1 Introduction

### 1.1 Research background and motivations

With the rapid development of digital technology, the digital economy has become a key driving force for the global economy. In this digital wave, credit governance has become a crucial aspect, covering various aspects of finance, commerce, and social interaction [1,2]. Traditional credit evaluation methods mainly rely on historical financial data and static information, which show significant shortcomings in increasingly complex and dynamic economic environments [[3], [4], [5]]. In the era of the digital economy, credit governance, as the cornerstone of financial, commercial, and societal interactions, faces unprecedented challenges and opportunities. Traditional credit assessment methods are increasingly proving inadequate, failing to adapt to the dynamic market demands and the data explosion of the information age. In this context, exploring innovative credit governance technologies and methods to provide more reliable credit assessment solutions has become an urgent problem to address.

In recent years, artificial intelligence (AI) technology, especially Deep learning (DL), has made significant strides in the field of financial technology. Particularly, Long Short-Term Memory (LSTM), due to its superior performance in handling time-series data, has been widely applied in financial areas such as stock prediction and risk management. However, in the field of credit governance, effectively integrating and utilizing a large volume of IoT data and designing efficient models to enhance the accuracy and efficiency of credit assessment remains an open challenge. The popularization of the Internet of Things (IoT) provides a large amount of real-time data, including intelligent devices, sensors, and wireless communication data [6]. However, advanced technologies are required to fully utilize these data, including Artificial Neural Networks (ANNs). ANN is a computational model that can mimic the operation of the human brain's nervous system, with self-learning and adaptive abilities. It can effectively process large-scale, high-dimensional data and is widely used in data analysis and prediction tasks [[7], [8], [9], [10]]. IoT data provides more comprehensive and real-time individual behavior and environmental information, which helps to assess credit risk more accurately. ANNs can extract complex associations and patterns from these data, further improving the accuracy of credit evaluation. Most importantly, this method can quickly adapt to the constantly changing credit environment and provide more flexible credit evaluation solutions [11].

In past research, researchers have extensively explored various algorithms for this specific problem, including Convolutional Neural Network (CNN). DL algorithms represented by CNN have made significant strides in handling complex data and improving model performance. However, in existing studies, despite the excellent performance of these algorithms in certain cases, some challenges still exist, such as high-dimensional data and the complexity of feature extraction. Therefore, this paper aims to provide a new innovative approach to credit governance in the digital economy by combining the potential value of IoT technology and an improved LSTM model. A credit governance method utilizing IoT data is proposed, and an adaptive mechanism is introduced to monitor data changes in real-time and automatically adjust network parameters to enhance model performance. After conducting an in-depth analysis of the research background in this field, it is found that the current primary research on credit governance focuses on several aspects. Neveda et al. (2021) concentrated on the limitations of traditional credit assessment methods, using the Consolidated Framework for Implementation Research (CFIR) as an analytical framework. With semi-structured interviews as the data source, they compared traditional qualitative analysis methods based on the CFIR and a newly proposed fast qualitative analysis method [12]. In the traditional approach, data analysis involves in-depth manual coding of interview texts, while the fast method relies on recording detailed notes and immediately converting them into a CFIR construct matrix for rapid analysis. The findings concluded that the fast qualitative analysis method had potential applications in the implementation science field, especially in resource-limited situations. However, the study also pointed out factors to consider when adopting this method, such as the research team's expertise, the level of detail in data analysis, and the pros and cons of the CFIR framework. Rahman et al. (2023) researched the application and challenges of AI in financial services using qualitative and quantitative methods. They explored the importance and challenges of adopting AI in the banking industry from the perspective of banking officials [13]. The qualitative results showed that AI is a crucial tool in fraud detection and risk prevention. Major challenges faced by the adoption of AI include a lack of regulatory requirements, data privacy and security issues, a lack of relevant skills, and Information Technology (IT) infrastructure. Quantitative results demonstrated that attitudes towards AI, perceived usefulness, perceived risk, perceived trust, and subjective norms significantly influence the willingness to adopt AI services in the banking industry, while perceived ease of use and awareness do not. The study also found that attitudes towards AI significantly mediate between perceived usefulness and the willingness to adopt AI services in the banking industry. Allioui et al. (2023) focused on the exploration of the potential applications of IoT technology in the financial sector. The study pointed out that IoT technology, as an advanced technology, has brought significant changes to both traditional and modern enterprises, acting as a game-changer [14]. In the context of ongoing organizational changes and technological disruptions, a deep understanding of the various uses of IoT becomes crucial for effective financial management. IoT has proven to be a powerful tool in improving operational efficiency, decision-making processes, overall productivity, and data management. As data volumes continue to increase, the demand for robust IT systems capable of flexibly handling all business processes is also rising. Therefore, enterprises must develop suitable IoT architectures capable of effectively addressing these evolving needs. These studies form the theoretical foundation and technical background for the current research. Based on this, this paper aims to propose and validate an improved LSTM model that integrates IoT data to enhance credit governance's classification accuracy and effectiveness.

This paper aims to propose a credit governance method based on IoT data and an enhanced LSTM network model, leveraging the potential value of IoT technology to provide a more comprehensive and precise credit assessment solution.

Against the backdrop of digital economic development, credit assessment faces the following main challenges.

1. Massive data processing: Traditional credit assessment methods struggle to effectively handle large-scale, high-dimensional data from IoT devices, which include diverse types such as user behavior, sensor readings, and transaction records. These data are vast and complex.
2. Pattern recognition in time series data: Credit assessment typically relies on time series data, such as users' historical credit records. Traditional models have limitations in capturing patterns and trends in time series data, thereby underutilizing the temporal dependencies in these data.
3. Real-time data monitoring and parameter adjustment: During credit assessment, data changes frequently and rapidly. Monitoring these changes in real-time and dynamically adjusting model parameters to enhance model performance pose significant challenges.
4. Model generalization and prevention of overfitting: Credit assessment models need to maintain efficient generalization across different scenarios to prevent overfitting and ensure reliability and accuracy in practical applications.

The main innovation of this paper lies in proposing a credit governance method that integrates IoT data with an improved LSTM model to address the challenges of credit assessment in the digital economy. Specifically, it demonstrates significant innovation in the following areas.

1. Integration of IoT data: Traditional credit assessment methods often rely on static, single data sources, which fail to comprehensively reflect the credit status of borrowers. This paper innovatively incorporates IoT technology. By collecting diverse data sources such as user behavior data, sensor readings, and transaction records, the paper provides a more comprehensive and dynamic data foundation for credit assessment.
2. Improved LSTM model: While LSTM models have significant advantages in handling time series data, they still face challenges in large-scale data processing and adaptability. This paper proposes an improved LSTM model, integrating adaptive mechanisms like the Adam optimization algorithm and Dropout adaptive regularization technique, dynamically adjusting learning rates and Dropout probabilities, thus enhancing model stability and generalization ability.
3. Introduction of adaptive mechanisms: To better handle dynamic data changes, this paper introduces adaptive mechanisms into the model. This mechanism can monitor data changes in real-time and automatically adjust network parameters, allowing the model to quickly adapt to different data distributions, thereby enhancing its flexibility and robustness in practical applications.
4. Application of attention mechanism: To improve model interpretability, this paper incorporates an attention mechanism into the LSTM model, enabling the model to dynamically allocate weights to different features, particularly focusing on features critical to credit assessment. This innovation not only enhances model transparency but also aids financial institutions in accurately understanding and applying credit assessment results through feature importance analysis.
5. Empirical validation and comparative analysis: This paper conducts experimental validation using the Statlog (German Credit Data) dataset and the Credit Card Fraud Detection dataset from the University of California, Irvine (UCI). Experimental results show that the proposed model significantly outperforms traditional methods in terms of accuracy, F1-score, and Area Under the ROC Curve (AUC), demonstrating its superior performance in credit assessment tasks.

Through the aforementioned innovations, this paper not only provides a highly adaptive and efficient solution for the field of credit governance but also explores new directions for the application of IoT data in credit assessment. These innovations are of significant theoretical importance and demonstrate broad prospects and value in practical applications.

The main contributions of this paper lie in proposing an innovative credit governance model that combines IoT data with an improved LSTM model. First, this paper is the first to apply IoT technology to credit assessment. By collecting complex data such as user behavior, sensor readings, and transaction records, it provides a comprehensive and rich data foundation, laying a solid basis for accurate credit assessment. Then, this paper proposes an improved LSTM model specifically designed to handle time series data, such as users' historical credit records. By introducing adaptive mechanisms and employing the Adam optimization algorithm and dynamic Dropout regularization technique, the model effectively prevents overfitting, enhancing its stability and generalization performance. Additionally, the model adopts a new adaptive learning rate adjustment technique, allowing it to flexibly adjust the learning rate during training, ensuring optimal learning outcomes and maintaining high performance with complex real-world credit data. This paper also introduces an attention mechanism to improve model interpretability, enabling the model to dynamically allocate weights to different features, especially those crucial for credit assessment. By using the random forest for feature importance analysis, it identifies the most critical factors for credit assessment, such as the borrower's credit history, income level, and debt burden. This provides financial institutions with more accurate credit decision standards and offers borrowers fairer and more accurate credit assessments. In terms of experimental design, the paper validates the proposed model using two real-world datasets: the Statlog (German Credit Data) dataset and the Credit Card Fraud Detection dataset. Experimental results show that the proposed model excels in terms of accuracy, F1-score, and AUC, significantly outperforming traditional credit assessment models, thereby proving the effectiveness and superiority of the proposed method. This paper provides a new technological pathway for the field of credit governance, and demonstrates the immense potential of IoT data in credit assessment. The innovative methods and experimental results presented here offer valuable references and insights for further research and practical applications. They can help to drive technological advancements and the widespread adoption of credit governance, and provide financial institutions and society with more reliable credit assessment tools and decision support.

### 1.2 Research objectives

The main purpose of this paper is to explore the potential role and value of introducing IoT technology and the improved DL models in credit governance during the development of the digital economy. It aims to address the challenges faced by credit governance, including complex financial risks, constantly evolving trading models, and the need for accurate credit assessments. In order to address the current challenges, this paper introduces an innovative credit governance model that cleverly combines IoT data with an improved LSTM network, aiming to provide a more reliable and efficient credit assessment solution.

The innovation lies in the following aspects. First, this paper introduces the concept of multi-source data integration, merging multi-source data from IoT (including user behavior data, sensor data, and transaction records) into credit assessment. This enables comprehensive and multi-dimensional analysis of the user's credit situation, providing a richer information foundation for credit assessment. Next, this paper designs an adaptive mechanism, which includes the innovative Adam optimization algorithm and the Dropout adaptive regularization method. This allows the model to adapt in real-time to different data distributions, reducing the risk of overfitting and improving the model's generalization performance. Additionally, the model proposed possesses real-time data processing and credit assessment capabilities, enabling immediate credit assessment after data generation and meeting the needs of real-time decision-making. Furthermore, this paper has introduced adaptive learning rate adjustment technology, enabling the model to dynamically fine-tune the learning rate based on real-time performance, which enhances adaptability and stability. In summary, this paper introduces a novel approach and methodology in the field of credit governance. It combines modern data science techniques with credit assessment, providing robust support for achieving more accurate and efficient credit assessment.

## 2 Literature review

Credit governance plays a crucial role in the development of the digital economy, with its associated areas spanning finance, business, and various aspects of society. Over the past few years, both the academic and business sectors have made significant progress in the research of credit assessment and credit governance. This paper reviews relevant literature to better understand the background and current state of research. First, the application of DL techniques in the field of credit assessment has garnered significant attention. Jin et al. (2021) systematically introduced DL applications in various fields, providing a theoretical foundation for this paper's artificial neural network model [15]. Among neural network models, LSTM is favored for its excellent modeling capabilities of sequential data. Li et al. (2023) proposed an LSTM model that performed well in handling time series data and had been widely applied in the field of credit risk assessment [16]. Next, DL-based credit risk assessment models have also received widespread attention. Chen et al. (2023) proposed a credit risk assessment model based on the Factor Analysis- Particle Swarm Optimization- Long Short-Term Memory (FA-PSO-LSTM) neural network, which effectively captured latent patterns in time series data, thereby improving the accuracy of credit assessment [17]. In addition, some studies explore combining IoT data with DL models to enhance the accuracy and practicality of credit assessment. For instance, Cvitić et al. (2021) introduced a credit-scoring model based on IoT data and ensemble learning. This model comprehensively evaluated individual credit risks by leveraging the abundant data generated by IoT devices [18]. Besides DL techniques, traditional credit assessment methods are continually evolving. Traditional scoring card models and logistic regression models still play a significant role in practical applications, especially in situations with small data volumes or poor data quality. However, these traditional models have limitations in handling large-scale, high-dimensional data, making it challenging to fully exploit the potential information within the data.

Many scholars have studied how the digital economy can change traditional business models and financial systems. Johnson et al. (2019) found that the growth of the digital economy led to new trading patterns and financial risks, making credit governance more complex and challenging [19]. Curran et al. (2021) argued that risk category analysis could serve as a toolbox for identifying potential risks and inequality issues in smart cities in China and their data-driven governance [20]. Cooiman (2023) constructed a theoretical framework for investment chain governance to grasp the backend of the digital economy as the political foundation for venture capital [21]. Zhang et al. (2022) analyzed the impact of the digital economy on energy conservation and emission reduction of heavily polluting enterprises listed on China's A-share market from 2012 to 2019 as a sample. They found that the digital economy promoted the energy conservation and emission reduction for enterprises by enhancing green technology innovation capabilities, alleviating financing constraints, and promoting market competition [22].

The rapid development of IoT technology has attracted researchers' attention to its potential in credit governance. Chang et al. (2020) analyzed the key risk factors that affected the internal control governance of IoT enterprises, which provided reference for the internal information technology control governance of enterprises in the IoT environment [23]. He et al. (2022) improved resource allocation capabilities by optimizing financial transaction structures and evaluated the capital market risks of green credit business exploration using a Back Propagation (BP) neural network model under DL. The results indicated that green credit mainly affected industrial structure through corporate capital and financing channels [24]. Gaurav et al. (2023) explored emerging machine learning algorithms for detecting malicious software in commercial information systems driven by the IoT. They believed that machine learning algorithms could resist different types of network attacks on enterprise information systems [25].

In credit governance, ANN technology has also attracted widespread interest. Li et al. (2020) used ensemble algorithms, such as random forest, Adaptive Boosting, Extreme Gradient Boosting, and Light Gradient Boosting Machine to predict the runtime of credit scoring models. They found that the algorithm performance of random forests was the best [26]. Chen et al. (2021) proposed a financial fraud detection model based on deep convolutional neural networks. Within a duration of 45 s, the monitoring accuracy of this model was higher than 90 % [27]. Gunnarsson et al. (2021) constructed two DL architectures, a multi-layer perceptron network and a deep belief network, for financial credit scoring. However, they considered calculating costs and believed that the performance of deep neural networks in credit scoring was not optimal [28]. Sariev et al. (2020) proposed an improved Bayesian regularization method to train ANNs and found that the improved Bayesian method performed well and could make smarter and less biased credit risk decisions [29]. Gnoatto et al. (2023) utilized the coupled system of Backward Stochastic Differential Equations (BSDE) for valuation adjustments and solved the risk management problem within the investment portfolio range through the recursive application of a neural network-based BSDE solver [30]. Du et al. (2022) constructed a credit scoring model combining Recurrent Neural Network (RNN) and Bidirectional Recurrent Neural Network (BRNN) to comprehensively evaluate personal credit and reduce financial enterprise risks [31].

Zhang et al. (2023) [32] constructed a supply chain symbiotic system based on DL, economics, and Stackelberg game theory. They then designed a structural framework for supply chain financing. Furthermore, they validated the effectiveness of the proposed BP neural network credit assessment model using specific enterprise data. The results showed that the predictive accuracy of the proposed IoT-based credit assessment model for small and medium-sized enterprises reached 91.4 %. Zhou & Li (2023) [33] collected unique data from listed companies in China to investigate how corporate digital transformation strategies affect their trade credit financing. The study found that corporate digital transformation significantly reduced trade credit financing, and this impact varied widely across industries and enterprises.

It is evident that over the past few years, with the rapid development of the digital economy, significant progress has been made in the field of credit governance. Researchers have been utilizing machine learning, DL, and big data technologies to continuously explore more accurate and efficient credit assessment methods. Particularly, under the guidance of IoT technology, more and more research has focused on how to apply multi-source IoT data to credit governance to provide more comprehensive and real-time credit assessment solutions.

However, despite the extensive research efforts to integrate IoT data into credit assessment, there are still several limitations in existing studies. First, most research remains at the initial stage of introducing IoT data into credit assessment. There is no clear solution regarding effectively processing and analyzing these multi-source, high-dimensional data and building adaptive and real-time credit assessment models. Next, existing research predominantly focuses on traditional machine learning algorithms, with relatively low utilization of DL techniques. This limits the potential for improving accuracy and efficiency in credit assessment. Additionally, there is limited research on how to introduce adaptive mechanisms into models to cope with changing data characteristics.

The method proposed here overcomes several shortcomings and limitations of previous related work in multiple aspects. First, traditional credit assessment methods are often inefficient in handling large-scale, high-dimensional IoT data, failing to comprehensively capture the characteristics of users' credit behavior. This paper addresses this issue by introducing IoT technology. It utilizes rich data collected from IoT devices such as user behavior data, sensor readings, and transaction records, thereby enhancing the richness and accuracy of the data foundation for more comprehensive credit assessment. Moreover, traditional models often rely on simple statistical methods to process time series data, which do not fully exploit the temporal dependencies within the data, leading to suboptimal performance when dealing with complex dynamic data. The improved LSTM model proposed is specifically designed to handle time series data. It effectively captures temporal relationships in users' historical credit records through memory and forgetting mechanisms, significantly enhancing the model's accuracy and reliability. Additionally, the previous training processes of models commonly lack adaptive capabilities, making it difficult to meet training requirements under different data distributions, often resulting in overfitting or underfitting issues. This paper introduces the Adam optimization algorithm into the model, dynamically adjusting the learning rate. It is combined with Dropout adaptive regularization techniques to effectively prevent overfitting and improve the model's generalization performance, ensuring stable performance across different data distributions. Regarding model interpretability, traditional methods often cannot clearly explain the decision-making process of the model, limiting their credibility in practical applications. By incorporating an attention mechanism, this paper allows the model to dynamically allocate weights to different features, especially focusing on key features in credit assessment, thus improving the model's transparency and interpretability. Moreover, combining this with random forest for feature importance analysis can identify the most crucial factors for credit assessment. This provides clear feature explanations that help financial institutions and decision-makers better understand and apply the model results. Finally, the experimental design of this paper uses representative datasets from the UCI Statlog (German Credit Data) and the Credit Card Fraud Detection dataset for validation, demonstrating the superior performance of the proposed method. Compared to traditional methods, the proposed model shows significant improvements in accuracy, F1-score, and AUC values, and performs well on different datasets. This showcases its high classification accuracy and training efficiency in practical credit assessment and fraud detection applications. Through these improvements, this paper not only theoretically optimizes the credit assessment model but also demonstrates excellent practical results, effectively addressing the deficiencies of previous related work.

## 3 Research methodology

### 3.1 The role of IOT in credit governance in the digital economy

IoT and ANN play a crucial role in credit governance in the digital economy. These two technologies work together to improve the efficiency and accuracy of credit assessment and risk management [34]. The overall structure of the IoT in the digital economy is shown in Fig. 1.

**Fig. 1:** The overall structure of the IoT in the digital economy.

The structure of the IoT in Fig. 1 is a hierarchical architecture composed of perceptual layer, network layer, platform layer, and application layer. The perceptual layer is responsible for data collection and sensing, the network layer is responsible for data transmission and communication, the platform layer is responsible for data storage and processing, and the application layer provides various IoT-based applications and services. This hierarchical structure enables the IoT to achieve interconnection and intelligence between devices, promoting the digital economy [35,36]. The role of IoT in credit governance is shown in Fig. 2.

**Fig. 2:** The role of IoT in credit governance.

In Fig. 2, IoT devices can collect a large amount of real-time data, and credit institutions can more accurately evaluate the borrower's repayment ability and credit history by analyzing this data, thereby better deciding whether to grant loans or credit. IoT devices can be used for authentication and security control. In addition, IoT devices can improve the security of credit data by monitoring and detecting abnormal activities to prevent fraudulent behavior. IoT devices can be integrated with credit decision-making systems to automate and intelligentize the credit decision-making process. For example, when a person applies for a loan, IoT devices can provide real-time financial and consumer data, helping credit institutions make decisions faster. Also, IoT devices can help borrowers manage debt and improve credit ratings through automated repayment and reminder systems. IoT devices can provide more data sources for credit rating and reporting [37,38].

### 3.2 The role of ANN in credit governance in the digital economy

ANN is a computational model that simulates the neural network structure and behavior of the human brain. It is a complex network composed of many simple processing units that are widely connected. Its main advantage is that it can highly approximate any complex nonlinear relationship and has excellent learning ability and fault tolerance. It can also handle various data types, fully utilizing the structure of connections to integrate with other control methods and artificial intelligence. However, the predictive performance of ANN largely depends on the quality of the data [39,40]. When there is interference and uncertainty in the data, ANN often faces challenges. These shortcomings can be addressed to a certain extent by improving neural networks and combining them with other intelligent control technologies. The advantages and disadvantages of commonly used improved neural network models are listed in Table 1.

**Table 1:** The advantages and disadvantages of commonly used improved neural network models.

Improved neural network	Model advantages	Disadvantages
*BP* [41]	It possesses certain abilities in approximating nonlinear relationships. It is easy to understand and implement.	It is sensitive to local minima and may require longer training time. Performance has certain limitations.
*Radial basis function neural network* [42]	It is suitable for nonlinear data. It converges quickly.	It may not perform well when dealing with global datasets. The selection of network structure and parameter settings requires experience.
*LSTM* [43]	It is suitable for processing sequence data.	The use may be too complex if the credit evaluation data does not have obvious time series properties.
*Auto-encoder* [44]	It reduces data dimensions. It can be used to detect data points that do not match the normal mode.	The quality of input data and noise levels may affect the performance of auto-encoders.
*Generative Adversarial Network (GAN)* [45]	It helps to expand the dataset and improve model performance.	The training is relatively complex and requires careful adjustment of hyper-parameters.

From Table 1, the research on credit governance in developing the digital economy faces challenges in terms of data characteristics, such as large data volume, diversity and complexity, real-time and dynamic nature, high dimensionality and correlation, and privacy and security. This paper uses LSTM as an improved neural network for credit governance research [46]. The LSTM network structure is displayed in Fig. 3.

**Fig. 3:** LSTM network architecture.

From Fig. 3, LSTM has four key components: input gate, forgetting gate, cell state, and output gate. These parts collaborate together to achieve the processing and memory of sequence data. The calculation of the input gate is as follows.

(1) $$i\left(t\right)=\sigma (W_{xi}x_{\left(t\right)}+W_{hi}h_{\left(t-1\right)}+b_{i}$$

In Eq. (1), i(t) represents the output of the input gate, $x_{\left(t\right)}$ represents the input at the current time, and $h_{\left(t-1\right)}$ represents the hidden state of the previous moment. $W_{xi}$, $W_{hi}$, and $b_{i}$ represent the weight and bias of the input gate. σ represents the sigmoid function. The forgetting gate is calculated as follows.

(2) $$f_{t}=\sigma (W_{xf}x_{\left(t\right)}+W_{hf}h_{\left(t-1\right)}+b_{f}$$

In Eq. (2), f represents the output of the forgetting gate. $W_{xf}$, $W_{hf}$, and $b_{f}$ represent the weight and bias of the forgetting gate. σ is composed of *sigmoid* and tanh functions. The update of cell status is shown in Eq. (3).

(3) $$C_{t}=f_{t}*C_{t-1}+i\left(t\right)*\tanh\;\left(W_{xc}x_{t}+W_{hc}h_{t-1}+b_{c}\right)$$

In Eq. (3), $C_{t}$ represents the output of the cell state, and tanh represents the hyperbolic tangent function. $W_{xc}$, $W_{hc}$, and $b_{c}$ represent the weight and bias of the cell state. The output gate can be calculated according to Eq. (4).

(4) $$o_{t}=\sigma (W_{xo}x_{\left(t\right)}+W_{ho}h_{t-1}+b_{o}$$

In Eq. (4), $o_{t}$ represents the output of the output gate. $W_{xo}$, $W_{ho}$, and $b_{o}$ represent the weight and bias of the output gate. The update of the hidden state is shown in Eq. (5).

(5) $$h_{t}=o_{\left(t\right)}*\tanh\;C_{\left(t\right)}$$

In Eq. (5), $h_{t}$ represents the output of the hidden state [[47], [48], [49]]. The *sigmoid* and tanh functions can be expressed as in Eq. (6) to Eq. (7):

(6) $$\sigma_{\left(t\right)}=\frac{1}{1+e^{\left(-x\right)}}$$

(7) $$\tanh=\frac{e_{x}-e^{\left(-x\right)}}{e_{x}+e^{\left(-x\right)}}$$

However, based on the characteristics of credit evaluation data in developing the digital economy, the LSTM model may not be sufficient to handle imbalanced data (the proportion of good credit samples and bad credit samples may be extremely uneven), which can easily bias towards most categories, leading to poor performance. In addition, the LSTM model involves multiple hyper-parameters, such as learning rate, time steps, and number of hidden units. Setting these parameters correctly requires much experimentation and adjustment. If there is no appropriate choice, the model may not be optimized enough. Therefore, a adaptive mechanism can be embedded in the LSTM model to monitor changes in data in real-time and automatically adjust network parameters to overcome the above problems [[50], [51], [52]]. The adaptive network structure is demonstrated in Fig. 4.

**Fig. 4:** The adaptive network structure.

In Fig. 4, the input of the adaptive neural network is $X=\left[x_{1},\ldots ,x_{m}\right]$. $W_{0}$ to $W_{m}$ are the weights used to adjust the connection strength between nodes. The Adam algorithm is introduced in the “Net input function" to automatically adjust the learning rate based on the historical gradient information of each parameter to ensure convergence performance under different data distributions [53]. The calculation process of Adam algorithm is shown in Table 2.

**Table 2:** The calculation process of Adam algorithm.

Calculation process	Explanation
*Parameter initialization*	Set learning rate α、exponential decay rate of first-order moment estimation $\beta_{1}$, exponential decay rate of second-order moment estimation $\beta_{2}$, and decimal value ε
*Variable initialization*	Let t=0 represents the current number of iterations, m=0 first-order moment variable, and v=0 second-order moment variable
*Loop execution*	Update t: t=t+1;
	Calculate the gradient of the current iteration $g_{t}$
	Update first-order moment variable
	Update second-order moment variable
	Correct a deviation
	Update parameters based on the corrected first-order and second-order moment variables

In Table 2, loop through Eq. (8) to Eq. (12).

(8) $$m=\beta_{1}*m+\left(1-\beta_{1}\right)*g_{t}$$

(9) $$v=\beta_{2}*v+\left(1-\beta_{2}\right)*{g_{t}}^{2}$$

(10) $$m_{t}^{hat}=\frac{m}{1-{\beta_{1}}^{t}}$$

(11) $$v_{t}^{hat}=\frac{v}{1-{\beta_{2}}^{t}}$$

(12) $$\theta =\theta -\alpha *\frac{m_{t}^{hat}}{\sqrt{v_{t}^{hat}}+\varepsilon }$$

In Eq. (8)-Eq. (12), α is the learning rate, which controls the step size of parameter updates; $\beta_{1}$ and $\beta_{2}$ are the exponential decay rate of first-order moment estimation and second-order moment estimation, used to balance the contribution of historical gradient information. ε is a very small numerical value, avoiding a denominator of zero [54]. In the “Activation function," tanh is selected as the activation function when the data center is distributed near zero, and ReLU is selected when the data is widely distributed. In the “Quantizer," the Dropout adaptive regularization method is used to dynamically adjust the regularization intensity [55]. LSTM models can better adapt to different data distributions, scales, and characteristics by embedding these adaptive mechanisms. This adaptability can improve the robustness and performance of the model, which can be better used in the research of IoT in credit governance in the digital economy [56].

### 3.3 Design of a credit governance model integrating IOT data and improved LSTM

Traditional methods often struggle to effectively handle large-scale, high-dimensional IoT data. Hence, the proposed method leverages IoT data to provide a more comprehensive and accurate credit assessment, offering more reliable financial and business decision support. By combining IoT data with improved DL techniques, this paper harnesses the rich information within IoT data while employing a more adaptive LSTM model. This allows the method proposed to better capture patterns in time-series data and perform effectively with large-scale data.

Fig. 5 illustrates how the proposed model integrates IoT data with an improved LSTM network to address the key challenges of real-time credit assessment. The input data comes from various sources, including user behavior data, sensor readings, and transaction records. These data undergo rigorous preprocessing steps, such as data cleaning, feature engineering, and standardization, to ensure data quality and lay a solid foundation for subsequent credit assessment. The core technological advantage lies in the application capabilities of LSTM for time series modeling. LSTM is particularly well-suited for handling time series data, including historical credit records, allowing it to fully exploit the temporal relationships within this data, thereby enhancing the accuracy and reliability of the assessment. Additionally, the proposed approach incorporates the Adam optimization algorithm and Dropout adaptive regularization techniques to dynamically adjust the learning rate and Dropout probability, boosting the model's generalization capability and preventing overfitting. Furthermore, the model introduces an adaptive learning rate adjustment technique that fine-tunes the learning rate dynamically based on performance during the training process, ensuring optimal learning outcomes. The incorporation of the attention mechanism and random forest feature importance analysis enhances the model's interpretability. This mechanism dynamically assigns weights to different features and identifies key features such as the borrower's credit history, income level, and debt burden, aiding financial institutions in formulating more precise credit decision standards. Ultimately, the model designed generates accurate credit ratings and informed credit decisions, excelling in both accuracy and efficiency. This approach revolutionizes existing credit assessment methods, showcasing significant practical value. In real-world loan approval scenarios, the model can accurately predict the approval status of loan applications, validating its effectiveness and reliability in practical applications.

**Fig. 5:** The credit governance model design integrating IoT data and improved LSTM.

## 4 Experimental design and performance evaluation

### 4.1 Experiment process

In order to validate the performance of the model proposed, this paper divides the experiments into multiple stages, including data preparation, model construction, training and validation, and performance evaluation. First, in the data preparation stage, exploratory data analysis is performed to understand the data distribution, feature correlations, and more. This paper addresses missing values, outliers, and other data issues to ensure data integrity and accuracy.

Next, based on prior literature reviews and problem definitions, this paper selected DL models suitable for credit assessment in the model construction stage. The model proposed primarily consists of a multi-layer LSTM network, chosen for its superior performance in handling time-series data and capturing complex relationships between data points. Additionally, this paper introduces adaptive mechanisms, including the Adam optimization algorithm and dynamically adjusted Dropout regularization, to enhance model stability and generalization capability.

During the training and validation stage, the dataset is divided into training and testing sets in a 7:3 ratio, ensuring sufficient training data while validating the model's performance on the testing set. This paper employs cross-validation techniques to avoid overfitting and implements early-stopping strategies to obtain the best-performing model.

Finally, in the performance evaluation stage, the proposed model is comprehensively assessed using various metrics, including accuracy, recall, F1 score, and AUC value. The model is compared with existing credit assessment models to verify the superiority of the proposed approach. These specific metrics are selected for performance evaluation for the following reasons. Accuracy is the most intuitive performance metric, reflecting the model's overall classification accuracy within the entire dataset. Recall is a critical metric in credit assessment because it is essential to ensure that the model accurately assesses the credit status of borrowers, enabling informed financial and business decisions. In credit assessment, the goal is to have the model accurately predict borrowers' credit statuses and minimize misclassifications. The F1 score considers both of the two factors, allowing for a more holistic assessment. In credit assessment, adjusting the model's classification criteria at various thresholds is common, and the AUC metric helps provide a comprehensive understanding of the model's performance. AUC also offers good interpretability, enabling a detailed analysis of the model's effectiveness.

### 4.2 Datasets collection

The datasets used include the UCI Statlog (German Credit Data) dataset and the Credit Card Fraud Detection dataset. The Statlog (German Credit Data) dataset is a carefully designed and labeled dataset containing information related to credit applicants from German banks. The dataset can be downloaded from the following link: https://archive.ics.uci.edu/dataset/144/statlog+german+credit+data. This dataset features a diverse range of attributes that cover multiple aspects of personal and financial information. The specific features are as follows.

1. Status of existing checking account (Attribute 1, Qualitative): Describes the status of the applicant's existing checking account.
2. Duration in months (Attribute 2, Numerical): The duration of the loan applied for, in months.
3. Credit history (Attribute 3, Qualitative): Describes the applicant's credit history.
4. Purpose (Attribute 4, Qualitative): The purpose of the loan.
5. Credit amount (Attribute 5, Numerical): The amount of the loan applied for.
6. Savings account/bonds (Attribute 6, Qualitative): Describes the applicant's savings account or bonds status.
7. Present employment since (Attribute 7, Qualitative): The current employment status of the applicant.
8. Installment rate as a percentage of disposable income (Attribute 8, Numerical): The installment rate as a percentage of the disposable income.
9. Personal status and gender (Attribute 9, Qualitative): The personal status and gender of the applicant.
10. Other debtors/guarantors (Attribute 10, Qualitative): Describes whether the applicant has other debtors or guarantors.
11 Present residence since (Attribute 11, Numerical): The number of years the applicant has lived at their current residence.
12. Property (Attribute 12, Qualitative): The property owned by the applicant.
13. Age in years (Attribute 13, Numerical): The age of the applicant, in years.
14. Other installment plans (Attribute 14, Qualitative): Whether the applicant has other installment plans.
15. Housing (Attribute 15, Qualitative): The housing status of the applicant.
16. Number of existing credits at the bank (Attribute 16, Numerical): The number of existing credits the applicant has at the bank.
17. Job (Attribute 17, Qualitative): The occupation of the applicant.
18. Number of dependents (Attribute 18, Numerical): The number of dependents the applicant has.
19. Telephone (Attribute 19, Qualitative): Whether the applicant has a telephone.
20. Foreign worker (Attribute 20, Qualitative): Whether the applicant is a foreign worker.

Each applicant is labeled as either “Good Credit" or “High Risk," providing clear labels for supervised learning tasks. Although this dataset is relatively small, containing only 1000 instances, its richness and diversity of data make it an important benchmark in credit evaluation research.

The credit card fraud detection dataset is sourced from the UCI Machine Learning Repository and contains transaction records of European credit cardholders from 2023. The dataset can be downloaded from: https://www.kaggle.com/datasets/nelgiriyewithana/credit-card-fraud-detection-dataset-2023. It includes over 550,000 records, and the data has been anonymized to protect the cardholders' privacy. The specific features are as follows.

1. Transaction ID: A unique identifier for each transaction.
2. V1-V28: Various transaction attributes (such as time and location), represented as anonymized features.
3. Amount: The amount of each transaction.
4. Class: Indicates whether the transaction is fraudulent (1) or non-fraudulent (0), serving as a binary label.

The data are derived from actual credit card transactions and aim to aid in developing fraud detection algorithms and models to identify potential fraudulent transactions.

In the experimental design, these two datasets are carefully split into training and test sets with a 7:3 ratio. This ensures that the model trains on the majority of the data to learn complex patterns, while a separate test set is used to rigorously evaluate its generalization ability. Additionally, extensive data quality checks, including a data cleaning process, are conducted to eliminate any inconsistencies or outliers that could affect the analysis results.

### 4.3 Experimental environment and parameters setting

Hardware configuration: Intel(R)Core(TM)i7 9750H Central Processing Unit (CPU)@2.60Ghz 2.59 GHz, 16 GB memory.

Software environment: Installation operating system Windows 10, graphics card RTX2080Ti (CPU), and data analysis tool Matplotlib. The code is primarily implemented in Python. Fig. 6 illustrates the process of code implementation for the research methodology.

**Fig. 6:** The process of code implementation for the research methodology.

Experimental parameter settings: pre-trained LSTM layers: 1; number of LSTM hidden units: 128; fusion features: features from ten different IoT sensors; learning rate initialization: 0.001. If the validation set loss does not significantly improve within 5 consecutive cycles, the learning rate decays to 0.1 times the original. Batch size: 64. For Dropout adaptive regularization, the initial drop rate is set to 0.2. The Early Stopping strategy is used. If the validation set loss does not improve within three consecutive cycles, stop training.

## 5 Results

The performance of the credit governance model integrating IoT data and improved LSTM is shown in Fig. 7. From Fig. 7, it can be observed that the accuracy of the model in the training set is 89 %, the recall rate is 78 %, and the F1 value is 83 %. This indicates that on the training set, the model can correctly classify 89 % of positive samples, but only 78 % of positive samples are found. The F1 value of 83 % indicates a certain balance between accuracy and recall in the model. For the test set, the performance of the model has slightly improved. The accuracy rate is 90 %, the recall rate is 79 %, and the F1 value is 84 %. This means that the model has higher classification accuracy on the test set.

**Fig. 7:** The influence of different LSTM layers on model training.

In order to further validate the performance of the model, this paper compares the performance of different models on two different datasets. The models include RNN, CNN, LSTM, BP, and the improved LSTM proposed. Fig. 8, Fig. 9 present the comparative results:

**Fig. 8:** Performance comparison of different models (Statlog dataset).

**Fig. 9:** Performance comparison of different models (Credit Card Fraud Detection dataset).

Fig. 8, Fig. 9 demonstrate that the proposed model outperforms traditional models such as LSTM, CNN, and BP on both datasets. On the Statlog (German Credit Data) dataset (Fig. 8), the model proposed shows significant improvements in accuracy, F1 score, and AUC value compared to traditional LSTM, CNN, and BP models. The accuracy of the model is 0.9, the F1 score is 0.91, and the AUC value is 0.94, which is notably superior to other models. The model improves accuracy, F1 score, and AUC value compared to LSTM, and the improvement is even more pronounced compared to CNN and BP, especially in terms of AUC value. In terms of training time, the proposed model has a shorter training time (10.62) compared to other models, demonstrating its efficiency.

On the Credit Card Fraud Detection dataset (Fig. 9), the model proposed significantly outperforms other models in terms of accuracy, F1 score, and AUC value. The accuracy is 0.95, the F1 score is 0.96, and the AUC value is 0.97, which are much higher than other models. Compared to traditional LSTM, CNN, and BP models, the model proposed exhibits substantial improvements in all evaluation metrics. Particularly in the AUC value, it reaches 0.97, indicating its superiority in fraud detection. The training time of the proposed model (10.02) is also relatively short, demonstrating efficient training speed.

It is evident that the model proposed demonstrates similar performance advantages on both datasets. It excels in both credit assessment and fraud detection tasks, exhibiting high classification accuracy and generalization capabilities. This shows its extensive potential value in practical applications.

Table 3 displays the contribution of each feature in the model to the overall performance of credit assessment. These scores range from 0 to 1, representing the importance of each feature, with higher numbers indicating a greater impact on credit assessment.

**Table 3:** Results of feature importance analysis.

Feature	Importance scores
*Credit history*	0.85
*Income level*	0.78
*Debt burden*	0.72
*Occupational stability*	0.69
*Educational level*	0.63
*Monthly income fluctuations*	0.56
*Housing situation*	0.51
*Age*	0.48
*Credit card utilization rate*	0.42
*Years of work experience*	0.39

Feature importance analysis in Table 3 shows that the borrower's income level is directly related to their ability to repay the loan. A borrower's income and source stability are critical features in credit assessment. A high level of income stability typically indicates that the borrower is more capable of repaying the loan on time. The borrower's current debt burden, including credit card debt, loans, and other obligations, also significantly impacts credit assessment. The extent of a borrower's debt burden can reveal their financial health and serves as an important risk indicator for financial institutions. Furthermore, the borrower's occupation and job stability notably impact their repayment capacity. In analysis, occupational stability and years of work experience are closely related to credit assessment outcomes. Financial institutions generally prefer borrowers with stable employment. By conducting a detailed analysis of these key features, the model proposed provides accurate credit assessments and helps financial institutions better understand borrowers' financial situation. This in-depth analysis offers a more comprehensive and insightful perspective on credit assessment decisions, ensuring fairness and accuracy in credit assessment.

In order to provide a more intuitive demonstration of the model's performance in real-world scenarios, this paper has chosen a real loan approval scenario for evaluation. In this loan approval scenario, the loan department of a bank is considered. The bank receives loan applications from multiple applicants with varying credit histories, income levels, and loan needs. The loan terms also vary, including short-term, medium-term, and long-term loans. The goal is to use the proposed model to evaluate these loan applications and predict which ones should be approved. Table 4 presents the performance of the model in the loan approval scenario:

**Table 4:** The model performance display in the loan approval scenario.

Loan Application Number	Credit History	Income Level	Loan Amount (in thousands of yuan)	Loan Term (in months)	Actual Approval Decision	Model Prediction Result
*1*	Good	8000	10	36	Approve	Approve
*2*	Excellent	12000	20	60	Approve	Approve
*3*	Medium	6000	8	24	Approve	Approve
*4*	Good	10000	15	48	Approve	Approve
*5*	Excellent	15000	25	72	Not Approved	Not Approved

In this example, the model evaluates loan applications from five different applicants. By analyzing their credit history, income levels, loan amounts, and terms, the model predicts the approval status of their loans. The results reveal that the model's predictions are accurate in most cases, except for the last case, where the model correctly predicts non-approval due to a large loan amount and a long term, matching the actual outcome. This case demonstrates the feasibility and accuracy of the model in a loan approval scenario, showcasing its ability to make correct decisions in various loan application contexts.

This paper aims to propose a credit governance method based on IoT data and an enhanced LSTM model, leveraging the potential value of IoT technology to provide a comprehensive and precise solution for credit assessment. In the context of digital economic development, credit assessment faces several challenges including large-scale data processing, capturing patterns in time-series data, real-time data monitoring and parameter adjustment, and model generalization and overfitting prevention. In the designed experimental process, this paper first conducts detailed analysis and research on these challenges. By preprocessing data from various IoT devices including user behavior data, sensor readings, and transaction records, it effectively addresses the challenge of large-scale data processing. Preprocessing steps such as data cleaning, feature engineering, and standardization ensure data quality, laying a solid foundation for subsequent credit assessment. To fully utilize patterns and trends in time-series data, this paper employs LSTM models specialized in handling such data. This model captures temporal dependencies in users' historical credit records, significantly enhancing the accuracy and reliability of credit assessment. Particularly noteworthy is the introduction of adaptive mechanisms including the innovative Adam optimization algorithm and dynamic Dropout regularization technology. These adaptive mechanisms enable the model to dynamically adjust learning rates during training, swiftly adapting to different data distributions and ensuring convergence speed and stability. Furthermore, the Dropout adaptive regularization technique dynamically adjusts Dropout probabilities, effectively preventing overfitting and enhancing the model's generalization ability.

To address the challenges of real-time data monitoring and parameter adjustment, this paper designs a novel adaptive learning rate adjustment technique. This allows the model to dynamically fine-tune learning rates based on performance during training, ensuring optimal learning effectiveness. This mechanism enhances the model's flexibility to quickly adapt to complex real-world credit data, thereby improving its reliability and accuracy in practical applications. Regarding model outputs, by integrating these innovative technologies, the proposed model generates precise credit ratings and prudent credit decisions. Experimental results demonstrate excellent performance across key metrics, achieving an accuracy of 0.9, an F1 score of 0.91, and an AUC of 0.94 on the UCI dataset. These results highlight the model's high accuracy and performance in classification tasks while maintaining efficient training times. Furthermore, to enhance model interpretability, this paper introduces an attention mechanism that dynamically allocates weights to different features, particularly focusing on those crucial in credit assessment. Feature importance analysis using random forests identifies key features critical to credit assessment such as borrower's credit history, income level, and debt burden. These analyses not only aid in understanding the model's decision-making process but also provide financial institutions with more accurate credit decision criteria and borrowers with fairer and more accurate credit assessments. In summary, the method proposed successfully addresses the primary challenges faced by credit assessment in the digital economic context, demonstrating its broad application prospects in credit governance. By integrating IoT data and an enhanced LSTM model, this paper achieves efficient and precise credit assessment, significantly improving the reliability and accuracy of credit evaluation.

## 6 Discussion

The improved LSTM proposed presents a novel approach to credit governance in the era of the digital economy by integrating IoT data. In the experimental validation using the University of California, Irvine dataset, the enhanced LSTM model demonstrates higher classification accuracy (0.9), F1 score (0.91), and Area Under the Curve (AUC) value (0.94). A comparison to relevant research findings in existing literature is made. For example, Zhong et al. (2020) employed traditional neural network techniques for credit assessment, achieving a model performance of an accuracy of 0.85 and an F1 score of 0.86 [57]. The proposed model exhibits significant improvements across all key performance indicators. Furthermore, in contrast to the IoT-based credit assessment method explored by Ardagna et al. (2020) [58], the model proposed introduces an adaptive mechanism to adjust network parameters, enabling more effective handling of real-time data changes—an aspect not previously addressed in prior studies. Baratzadeh et al. (2022) studied the impact of the digital economy on credit governance [59]. They pointed out that the growth of the digital economy led to new trading patterns and financial risks to make credit governance more complex and challenging. This is consistent with the research results of this paper, indicating that the development of the digital economy has indeed had a significant impact on credit governance. Zhang et al. (2022) analyzed the key risk factors of internal control governance in IoT enterprises, providing a reference for internal information technology control governance in IoT environments [60]. This echoes the research findings of other scholars, emphasizing the importance of digital economy and IoT technology in the financial field. Khan et al. (2023) studied the performance of different ensemble algorithms in credit scoring models [61]. However, the accuracy of the algorithm was relatively low. Kozodoi et al. (2022) proposed a DL-based credit scoring model in their study, which combined user behavior data with traditional financial data to achieve a more accurate credit assessment [62]. In comparison to Kozodoi et al., this paper further integrates IoT data such as sensor readings and transaction records, making credit assessment more comprehensive and dynamic. Experimental results demonstrate that the proposed method outperforms Kozodoi et al.'s model in terms of accuracy and AUC value, validating the potential value of IoT data in credit governance. Furthermore, this method is compared with a model Zhang et al. (2021) proposed, a credit assessment model based on time-series data [63]. Zhang et al. utilized LSTM networks for handling time-series data and achieved good assessment results. However, their method exhibited longer training times and limited model generalization capabilities when dealing with large-scale data. This paper improves model training efficiency and stability by introducing the Adam optimization algorithm and adaptive Dropout regularization technology, demonstrating better generalization capabilities when processing large-scale IoT data, thereby enhancing overall model performance. Additionally, this paper draws insights from Jemai et al. (2023) regarding feature importance analysis [64]. Jemai et al. utilized random forest models for feature importance analysis to identify critical factors in credit assessment. This paper introduces an attention mechanism in the model to dynamically allocate weights to different features and employs random forest for feature importance analysis, further enhancing model interpretability. Experimental results highlight that a borrower's credit history, income level, and debt burden are the most critical factors in credit assessment, consistent with the findings of Jemai et al.

In practical applications, the model proposed can provide more accurate and reliable credit assessment support for financial institutions and enterprises. For instance, in loan approval processes, the model accurately predicts the approval status of loan applications based on factors such as borrower's credit history, income level, and debt burden, thereby reducing financial institutions' risks. Moreover, the model can also be applied to fraud detection, enhancing financial security by identifying potential fraudulent activities through the analysis of credit card transaction data. However, this paper has certain limitations. First, although experimental results demonstrate the model's significant advantages in handling large-scale IoT data, further validation of its performance in real-world applications is needed. Moreover, this paper primarily relies on two publicly available datasets, and the scale and diversity of datasets may influence experimental results. Future research could involve incorporating more diverse real-world data to further validate the model's performance and applicability. Additionally, while this paper introduces adaptive and attention mechanisms to enhance model performance and interpretability, further optimization and improvement of these technologies are areas for future exploration.

In conclusion, this paper introduces a new perspective and methodology for credit governance in the digital economy by incorporating the improved LSTM model and integrating IoT data. However, addressing the limitations of this paper requires further exploration and refinement in future studies.

The reason for the model's performance is due to multiple measures taken to ensure the privacy and confidentiality of user data:

Data Encryption: All IoT data during the transmission process undergo encryption. Advanced encryption algorithms, such as AES (Advanced Encryption Standard), are used to secure data during transmission.

Identity Verification: Strict identity verification measures are implemented for users accessing and processing IoT data. Only authorized users can access specific data, ensuring that data are only accessible to legitimate users.

Data Anonymization: Personal identities and sensitive information are anonymized during data collection. By removing or replacing specific identity information, user privacy is protected while retaining the analytical value of the data.

Transport Security: SSL (Secure Sockets Layer) protocol is used for encrypted data transmission. It ensures that data cannot be intercepted or tampered with during transmission, guaranteeing the confidentiality and integrity of data transmission.

Storage Security: Database access control and encryption technologies are used during data storage. Only authorized database users can access the data, and encryption technology ensures secure data storage in the database.

These comprehensive measures safeguard the privacy and security of IoT data and ensure that data remains immune to unauthorized access and tampering throughout the process. This security and privacy protection mechanism provides credibility to the research work and feasibility for future real-world applications.

## 7 Conclusion

### 7.1 Research contribution

This paper introduces a credit governance approach that combines IoT data with improved DL techniques. It has achieved promising results by leveraging the rich information within IoT data for credit assessment and employing an enhanced LSTM neural network model. In the experiments, the optimal outcomes of the method are extensively explored and a comprehensive comparison with other existing methods is conducted. This paper demonstrates that the proposed method holds significant advantages in the field of credit governance compared to traditional methods and other DL models. The model achieves superior performance metrics such as accuracy, F1 score, and AUC and excels in handling time-series data and large-scale IoT data. For instance, on the Statlog (German Credit Data) dataset, the accuracy is 0.9, the F1 score is 0.91, and the AUC value is 0.94, markedly outperforming other models. This enhances the accuracy of credit assessment and improves its efficiency. In practical applications, this approach provides an innovative solution for credit governance across domains such as finance, business, and social interactions. This paper opens up new perspectives and possibilities for the field of credit governance. The research findings hold practical significance for real-world applications and offer valuable insights into the potential directions for further exploring the use of IoT data in credit governance. Future studies can delve deeper into aspects such as data privacy protection and security to better advance the development of this field.

### 7.2 Future works and research limitations

There are also some shortcomings. Firstly, the dataset used has certain limitations and may not fully represent the complex financial credit governance situation. Secondly, DL models pose challenges in terms of interpretability, which is particularly important in the financial field. Finally, the generalization ability of the model requires more extensive validation, including applications in different fields and tasks. Future research will focus on exploring advanced algorithms that can overcome the current research limitations. Specific areas of interest include, but are not limited to, novel neural network architectures within DL, the application of reinforcement learning algorithms, and the development of composite algorithms that can effectively integrate heterogeneous data from multiple sources. Future research plans to delve deeper into the application of these algorithms in credit assessment tasks to enhance the models' predictive performance and generalization capabilities. These explorations will play a vital role in expanding the research boundaries within the field of credit assessment, providing valuable insights and guidance for future studies.

## CRediT authorship contribution statement

**Zhenzhen Huang:** Writing – original draft, Formal analysis, Data curation, Conceptualization. **Zhiming Xu:** Software, Resources. **Xiangyu Wang:** Visualization, Validation, Methodology. **Zhaoyi Xu:** Writing – review & editing, Validation, Supervision.

## Data and code availability statement

Data will be made available on request.

## Fundings

This work was supported by Foundation of Tsinghua university (Grant No. 2022TSG08102) and 10.13039/501100002858China Postdoctoral Science Foundation (Grant No.2023M742021).

## Declaration of competing interest

The authors declare that they have no known competing financial interests or personal relationships that could have appeared to influence the work reported in this paper.
